# Evaluation of Pelvic Floor Dysfunction by Pelvic Floor Ultrasonography after Total Hysterectomy for Cervical Cancer

This article has been retracted.

**DOI:** 10.1155/2022/5914344

**Published:** 2022-09-28

**Authors:** Dan-dan Liu, Jing Xin, Wei Liu, Yan-feng Zhang, Peishan Li

**Affiliations:** ^1^Obstetrics and Gynecology Department, Laishan Branch of Yantai Yuhuangding Hospital, Yantai, Shandong 264003, China; ^2^Obstetric Center, Qingdao Eighth People's Hospital, Qingdao, Shandong 266000, China; ^3^Health Management Division, Qingdao Eighth People's Hospital, Qingdao, Shandong 266000, China; ^4^Surgery, Laishan Branch of Yantai Yuhuangding Hospital, Yantai, Shandong 264003, China; ^5^Operation Room, Laishan Branch of Yantai Yuhuangding Hospital, Yantai, Shandong 264003, China

## Abstract

**Objective:**

To study the value of pelvic floor ultrasonography in evaluating pelvic floor dysfunction (PFD) after total hysterectomy for cervical cancer.

**Methods:**

All the enrolled patients were given 4D pelvic floor ultrasound examination before and after surgery. The results of ultrasonic examination and the parameters of four-dimensional ultrasonic examination before and after surgery were analyzed, and the quality of life of the patients before and after surgery was evaluated.

**Results:**

Postoperatively, the posterior angle of bladder and urethra, the rotation angle of urethra, the decreased value of bladder neck, and the distance between bladder neck and pubic symphysis were (122.60 ± 9.53)°, (136.47 ± 14.67)°, (58.90 ± 18.19)°, (18.14 ± 7.32) mm, and (2.76 ± 0.46) cm, significantly greater than the preoperative (89.90 ± 9.59)°, (107.30 ± 9.96)°, (27.59 ± 10.96)°, (13.27 ± 5.69) mm, and (2.24 ± 0.21) cm (*P* < 0.05). Postoperative detrusor muscle thickness, bladder neck movement, residual urine volume, and bladder rotation angle (4.48 ± 0.82) mm, (0.64 ± 0.17) cm, (12.82 ± 2.69) ml, (12.11 ± 2.43)° were significantly higher than those of preoperative (3.70 ± 0.64) mm, (0.43 ± 0.18) cm, (4.83 ± 1.07) ml, (4.30 − 1.19)° (*P* < 0.05). The scores of emotional function, psychological function, social function, and physiological function were (2.35 ± 0.75) points, (2.45 ± 0.66) points, (2.30 ± 0.77) points, and (2.19 ± 0.71) points, significantly higher than those of (1.01 ± 0.50) points, (1.25 ± 0.54) points, and (1.00 ± 0.57) points before surgery, (1.05 ± 0.46) (*P* < 0.05).

**Conclusions:**

The application of pelvic floor ultrasonography to detect pelvic floor dysfunction after total hysterectomy can clearly display the anatomical structure of the pelvic floor, which is conducive to disease prevention and treatment. Four-dimensional pelvic floor ultrasound can clearly show the postoperative pelvic floor function, which is worthy of clinical promotion and reference.

## 1. Introduction

Cervical cancer (CC) is one of the most common gynecological malignant tumors, and its incidence is second only to breast cancer and currently ranks second in the global gynecological malignant tumors, which seriously threatens women's life and health. According to statistics, one-third of the total number of global cases happened in China each year [1]. At the same time, with the increase of HPV infection rate, the incidence of cervical cancer increases significantly and gradually tends to be younger. The current treatment of cervical cancer is based on the International Federation of Gynecology Obstetrics (FIGO) staging with the options of operation in the early stage, such as extensive hysterectomy plus pelvic lymph node dissection [2, 3]. As the number of cancer survivors continues to increase, the quality of life (QOL) of these survivors is an important consideration for healthcare providers, such as pelvic floor dysfunction [4]. In recent years, with the development of 3D multisection and 4D dynamic image acquisition techniques and their powerful data postprocessing capacity, pelvic floor ultrasound has begun to be applied in clinical practice. The 4D view off-machine analysis can be exploited to reconstruct 3D plane image, measured in the corresponding physiological action state with easy operation, reliable inspection data, and low cost [5]. However, there are few studies on the effect of 4D pelvic floor ultrasound in the diagnosis of pelvic floor function after cervical cancer surgery. We hypothesized that four-dimensional pelvic floor ultrasound can be complementary or alternative route to improve the comprehensive diagnosis of the extent of anatomical structure of the pelvic floor.

### 1.1. Patients

A total of 119 patients who underwent hysterectomy cervical cancer surgery in our hospital from January 2019 to August 2020 were identified as potential candidate, including 68 patients with stage I cervical cancer and 51 patients with stage II cervical cancer. The ethics committee of the hospital recorded this study; all patients acknowledged the purpose and the procedures of this research and signed informed consent.

### 1.2. The Inclusion Criteria

(1) Mean age was (52.87 ± 3.82) years (range 42-67) years; (2) mean body mass index was (22.60 ± 0.91) kg/m^2^. (3) 12weeks after surgery (4) without symptom of pelvic organ prolapses or history of pelvic surgery in the past (5) no other related treatments were received after surgery (6)have ultrasound examinations before and after surgery.

### 1.3. The Exclusion Criteria

(1) Patients with hypertension liver and kidney dysfunction and other serious underlying diseases. (2) Patients with a history of pelvic surgery, urinary surgery, nervous system, and infectious diseases. (3) Those patients who did not agree to participant in this study.

## 2. Methods

The ultrasonic images were collected using a GE Voluson E8 Color Doppler Ultrasound Machine equipped with RIC 5–9-D Probes. The working frequency was 5 to 10 MHz. 4D View 10.0 camera analysis software was used to reconstruct the data, and the instrument was set to pelvic floor ultrasound examination. Prior to the image collection, feces of the patients must be removed. The amount of residual urine in the bladder must be about 50 mL. The volume probe was outsourced to sterile protective sleeve, which was coated with disinfectant and chelating agent on both the inside and outside. The probe was firmly placed in the perineum of the patient to store the images including the midsagittal plane of the urethra, vagina, bladder neck, rectal junction, and pubic symphysis. The angle of urethral rotation, the vertical distance between the bladder neck and the lower symphysis pubis (BSD), the degree of bladder neck depression (BND), and the posterior horn of bladder and urethral angle were also measured at both the resting and maximum Valsalva action state. The reference value of the posterior angle of the bladder and urethra is 90° to 120°, and the reference value of the urethral rotation angle is 30° to 45°. All detections were repeated 3 times.

### 2.1. Diagnostic Criteria

Stress urinary incontinence diagnostic criteria: (1) BND ≥ 2.0 cm in the maximal Valsalva state; the posterior angle of the bladder and urethra ≥ 120° and the bladder neck rotation angle ≥ 20° in the maximal Valsalva state; (2) caused by sneezing, coughing, and laughter urine overflow occurs when there is increased pressure in the abdomen. The diagnostic criteria for pelvic organ prolapse are: the vertical distance between the lowest point of the pelvic organ and the lower part of the pubic symphysis detected by ultrasound of the perineal pelvic floor is greater than 1 cm. The posterior angle of the bladder and urethra is greater than or equal to 140°, and the rotation angle of the urethra is less than 45°. Combined with the changes in the anatomical structure of the pelvic floor, clinical manifestations, and the characteristics of this transperineal four-dimensional pelvic floor ultrasound imaging, the results were obtained. The four-dimensional pelvic floor ultrasound was used to detect stress urine. Four items of incontinence, bladder prolapse, uterine prolapse, and rectal prolapse were used as diagnostic indicators. The comparison of four-dimensional pelvic floor ultrasound examination parameters of pelvic floor dysfunction after cervical cancer hysterectomy in different states uses SF-36 to evaluate the quality of life [6]. SF-36 includes four aspects: emotional function, mental function, social function, and physiological function. According to the severity of the impact of symptoms on daily life, patients are divided into no effect (0 points), mildly affected (1 point), moderately affected (2 points), and severely affected (3 points), the higher the score, the worse the quality of life.

### 2.2. Statistical Analysis

Statistical analysis was performed using SPSS 23.0 software. Continuous data were expressed as mean ± standard deviation, group *t*-test was used for comparison between two groups. Chi-square test was used for the comparison of binary data. Multiple logistic regression analyses were conducted to identify the potential risks. In this present study, *P* < 0.05 was considered that the differences were statistically significant.

### 2.3. Results of Four-Dimensional Pelvic Floor Ultrasound Diagnosis

Among 119 patients with cervical cancer who underwent hysterectomy, 57 cases (47.90%) of bladder prolapse were found by four-dimensional pelvic floor ultrasonography, 22 cases (18.49%) of rectal prolapse, 7 cases (5.88%) of uterine prolapse, and 33 cases (27.73%) of stress urinary incontinence.

### 2.4. Comparison of Parameter Values of Four-Dimensional Ultrasonography before and after Surgery

After surgery, urinary tract rotation angle, the vertical distance between the bladder neck and the pubic symphysis (BSD), the bladder neck reduction (BND) in the resting state and the posterior angle of the bladder and urethra in the maximum Valsalva state were significantly higher *t* (*P* < 0.05).As shown in Table 1.

### 2.5. Changes of Lower Urinary Tract in Patients before and after Surgery

As shown in Table 2, the degree of bladder neck motion, bladder residual urine volume, bladder rotation angle, and bladder detrusor thickness were significantly improved after surgery (*P* < 0.05).

### 2.6. Comparison of the Quality of Life of the Two Groups of Patients before and after Surgery

As shown in Table 3, the scores of the patients after operation were higher than before operation (*P* < 0.05), that means the quality of life after operation was worse.

## 3. Discussion

From the perspective of human anatomy, the female pelvic cavity involves the cervix, uterus, and supporting tissues, as well as part of the pelvic lymph nodes and vagina, which can play important role in undertaking and supporting to ensure the normal state of pelvic organs [7]. Pelvic floor dysfunction can lead to pelvic floor dysfunction diseases such as stress urinary incontinence and pelvic organ prolapse. According to research reports, childbirth and surgery are the main causes of pelvic floor dysfunction. The hysterectomy not only needs to cut off the main and sacral ligaments in the center of the pelvic floor but also needs to push down the bladder and rectum, which causes about 20% patients have symptoms of urinary and stool disorders and incontinence [8].

At present, the clinical methods for evaluating the structural and functional changes of the female pelvic floor mainly include clinical staging, urodynamic examination, and acupressure test, while the imaging methods used for the examination of female pelvic floor dysfunction mainly include CT, ultrasound, and nuclear magnetic resonance [9]. Although MRI technology has high contrast resolution and good impact space, it is difficult to repeat observation due to its high cost, long inspection time, and cannot dynamically observe pelvic function. CT is difficult to be accepted by patients because of its radiation, ultrasound because of its minimally invasive, nonradiation, dynamic observation, and other characteristics, it is widely used in clinical examination and diagnosis [10, 11]. Four-dimensional pelvic floor ultrasound is a new inspection method, which is real-time dynamic imaging based on three-dimensional ultrasound [12]. Clinical studies have shown that four-dimensional pelvic floor ultrasound for pelvic floor dysfunction can dynamically observe the three-dimensional image of the pelvic floor and pelvic floor muscles in real time through three-dimensional stereo imaging, making up for the insufficiency of two-dimensional plane ultrasound, making clinical diagnosis more intuitive and the results more accurate. Exactly [13], the results of this study showed that the urinary tract rotation angle, bladder neck reduction (BND), vertical distance (BSD) between the bladder neck and the pubic symphysis, and the retro vesicourethral angle in the resting state and the maximum Valsalva state were significantly higher than those in the postoperative patients. Before surgery, the degree of bladder neck motion, bladder rotation angle, bladder residual urine volume, and bladder detrusor thickness were significantly greater than those of before surgery. This indicates that after hysterectomy, the uterine ligament and uterosacral ligament are cutoff and the bladder and rectum are pushed down, which will affect the innervation of the bladder and rectum, resulting in changes in the anatomical and physiological structure of the pelvic floor, resulting in pelvic floor dysfunction [14]. Although female pelvic floor dysfunction does not endanger the patient's life, it will seriously affect the patient's quality of life, and will have a negative impact on society, psychology, and daily life [15, 16]. Researchers compared the quality of life of patients with gynecological malignant tumors and postoperative benign uterine disease found that the symptoms of postoperative pelvic floor dysfunction in patients with malignant tumors were significantly higher than those in the control group. Our research data also showed that the quality of life of patients after surgery was worse.

In conclusions, cervical cancer patients are more likely to develop pelvic floor dysfunction after hysterectomy. Clinical medical workers should take four-dimensional pelvic floor ultrasonography to reduce the occurrence of pelvic floor dysfunction and improve the quality of life of patients.

## Figures and Tables

**Table 1:** Comparison of parameter values of four-dimensional ultrasonography before and after surgery ($\bar{X}\pm s$).

Group	*n*	BSD (cm)	BND (mm)	URA (°)	PUVA resting (°)	PUVA Valsalva (°)
Pre	119	2.12 ± 0.32	13.24 ± 5.59	27.58 ± 10.99	89.89 ± 9.61	107.27 ± 9.94
Post	119	2.76 ± 0.54^∗^	18.18 ± 7.32^∗^	58.90 ± 18.22^∗^	122.62 ± 9.51^∗^	136.42 ± 14.65^∗^
*t*		11.123	5.851	16.057	26.408	17.962
*P*		≤0.001	≤0.001	≤0.001	≤0.001	≤0.001

^∗^ *P* < 0.05.

**Table 2:** Changes of lower urinary tract in patients before and after surgery ($\bar{X}\pm s$).

Group	*n*	BNM (cm)	RBV (mL)	BRA (°)	DWT (mm)
Pre	119				
Post	119	0.43 ± 0.18	4.83 ± 1.07	4.30 ± 1.19	3.70 ± 0.64
*t*		0.64 ± 0.17^∗^	12.82 ± 2.69^∗^	12.11 ± 2.43^∗^	4.48 ± 0.82^∗^
*P*		9.253	30.107	31.488	8.180
		≤0.001	≤0.001	≤0.001	≤0.001

^∗^ *P* < 0.05.

**Table 3:** Comparison of the quality of life of the two groups of patients before and after surgery ($\bar{X}\pm s$).

Group	*n*	Emotion function	Mental function	Social function	Physiological function
Pre	119				
Post	119	1.02 ± 0.52	1.20 ± 0.52	1.20 ± 0.58	1.00 ± 0.52
*t*		2.34 ± 0.76^∗^	2.42 ± 0.71^∗^	2.38 ± 0.81^∗^	2.18 ± 0.74^∗^
*P*		16.637	15.122	12.921	14.232
		≤0.001	≤0.001	≤0.001	≤0.001

^∗^ *P* < 0.05.

## Data Availability

The data used to support the findings of this study are available from the corresponding author upon request.
